The article "[6]-Gingerol Inhibits Chikungunya Virus Infection by Suppressing Viral Replication" was published in 2021. Journal: Biomed Res Int.

# [6]-Gingerol Inhibits Chikungunya Virus Infection by Suppressing Viral Replication

**DOI:** 10.1155/2021/6623400

**Published:** 2021-03-27

**Authors:** Rahma F. Hayati, Cynthia D. Better, Dionisius Denis, Amalina G. Komarudin, Anom Bowolaksono, Benediktus Yohan, R. Tedjo Sasmono

**Affiliations:** ^1^Eijkman Institute for Molecular Biology, Ministry of Research and Technology/National Agency for Research and Innovation, Jl. Diponegoro 69, Jakarta 10430, Indonesia; ^2^Faculty of Pharmacy, University of Strasbourg, 4 Rue Blaise Pascal, Strasbourg 67081, France; ^3^Cellular and Molecular Mechanisms in Biological System Research Group, Department of Biology, Faculty of Mathematics and Natural Sciences, Universitas Indonesia, Depok, West Java, Indonesia

## Abstract

Chikungunya (CHIK) is a reemerging arboviral disease caused by chikungunya virus (CHIKV) infection. The disease is clinically hallmarked by prolonged debilitating joint pain. Currently, there is no specific antiviral medication nor commercial vaccine available for treatment of the disease, which makes the discovery or development of specific anti-CHIKV compounds a priority. Ginger (*Zingiber officinale* Roscoe) is widely known for its various health benefits. The compound [6]-gingerol is the main active ingredient found in ginger. This study sought to determine the potential of [6]-gingerol antiviral activity against CHIKV infection using *in vitro* human hepatocyte HepG2 cells. The antiviral activity mechanism was investigated using direct virucidal and four indirect (pre-, post-, full-, and prevention) treatment assays. [6]-Gingerol showed weak virucidal activity but significant indirect antiviral activity against CHIKV through post- and full treatment with IC_50_ of 0.038 mM and 0.031 mM, respectively, without showing cell cytotoxicity. The results indicated that [6]-gingerol inhibits CHIKV infection through suppression of viral replication. Together, this study confirms the potential use of [6]-gingerol for CHIK antiviral compound.

## 1. Introduction

Chikungunya (CHIK) is an acute febrile illness caused by infection with chikungunya virus (CHIKV). Firstly isolated in Tanzania in 1952, CHIKV has spread mainly in tropical and subtropical regions where appropriate vectors are prevalent [1]. The reemergence of the virus in East Africa, India, and around the Indian ocean in 2004-2007 caused a massive outbreak with significant economic impacts [2]. In Indonesia, CHIKV was firstly reported in Sumatera in 1982 which then spread to other major islands [3, 4]. Sporadic outbreaks have been reported in Java in 2000-2002, as well as recent detection of other provinces [4–6].

The virus, which belongs to the *Alphavirus* genus in the family of *Togaviridae*, is transmitted to humans by the bite of infected *Aedes* sp. mosquitoes. The CHIKV genome consists of 11.8 kb positive single-stranded RNA with two reading frames encoding four nonstructural proteins (NS1-NS4) in the first 5′ open reading frame and three structural (Capsid, E1, and E2) and two other proteins (E3 and 6K) in the second 3′ reading frame [7]. Phylogenetically, the virus has been classified into three distinct genotypes, namely, the West African, East Central, and South African (ECSA), and Asian genotypes [8].

The article "[6]-Gingerol Inhibits Chikungunya Virus Infection by Suppressing Viral Replication" was published in 2021. Journal: Biomed Res Int.

The clinical symptoms of CHIK, which share great similarity with dengue, include fever, headache, rash, and myalgia with debilitating arthralgia as the hallmark of CHIKV infection [9]. Although CHIK has a lower fatality rate compared to similar arboviral disease such as dengue, the inconvenience caused by CHIKV infection greatly affects one's daily life as the crippling joint pain persists for quite a long period [10]. Currently, CHIK's treatments are only symptomatic with no specific antiviral medicine available. In addition, commercial vaccines are also unavailable in the market although several potential CHIKV vaccine candidates are now in the clinical stages of development [11]. Therefore, it is important to find an effective treatment to avoid the daily life-inconvenience caused by the disease, besides preventive measure such as controlling mosquito population.

Ginger (*Zingiber officinale* Roscoe), a plant whose rhizome is widely used in Asia as a spice and as a component in traditional herbal medicine, has been shown to have multiple health benefits [12]. A number of studies have demonstrated that the plant possesses biological activities such as antioxidant, anti-inflammatory, antimicrobial, and anticancer effects [13–16]. In addition, ginger has also been reported to potentially prevent and manage obesity, diabetes mellitus, respiratory disorders, neurodegenerative diseases, and cardiovascular disease [17–21].

The compound [6]-gingerol is one of the major pharmacologically active constituents of ginger [12]. It is responsible for the pungent taste of fresh ginger caused by the presence of aromatic ketones in its chemical structure (Figure 1) [22]. This nonvolatile molecule possesses a favorable toxicity profile and various biological activities, such as antioxidation, anticancer, analgesic effect, and anti-inflammatory effects [23].

Here, we examine the antiviral activity of [6]-gingerol against CHIKV infection *in vitro* using HepG2 cells. We also sought to understand the mechanism of inhibition by comparing the different treatment assays. The findings may provide new insights on the use of [6]-gingerol in the management of CHIK disease.

The article "[6]-Gingerol Inhibits Chikungunya Virus Infection by Suppressing Viral Replication" was published in 2021. Journal: Biomed Res Int.

## 2. Material and Methods

### 2.1. Cell Lines and Virus

All cells used were originally obtained from American Type Culture Collection (ATCC) and have been maintained in Eijkman Institute's cell repository. The human (*Homo sapiens*) hepatocyte HepG2 cell line and Syrian baby hamster's (*Mesocricetus auratus*) kidney BHK-21 cell line were maintained in RPMI medium supplemented with 10% Fetal Bovine Serum (FBS), 1% antibiotic/antimycotic, and 2 mM of l-glutamine (all from Gibco-Thermo Fisher Scientific). The monkey kidney Vero (CCL81) cell line was maintained in MEM medium supplemented with 5% of FBS, 1% antibiotic/antimycotic, and 2 mM of l-glutamine (Gibco-Thermo Fisher Scientific). All cell lines were maintained at 37°C with 5% CO_2_ supplementation.

CHIKV strain JMB-192 (designated as CHIKV-JMB-192), isolated from a febrile patient in Jambi in 2015, has been characterized as an Asian genotype [6]. The virus was propagated in Vero-CCL81 and harvested when cytopathogenic effect (CPE) was observed in 70-80% of cells. Virus titer was measured by standard plaque assay on BHK-21 cells adapted from a DENV assay [24]. Briefly, 2 × 10^5^ cells/well were seeded in 24-well plates followed by incubation at 37°C under 5% CO_2_ for two days. Tenfold serial dilutions of CHIKV were added to the cells for 1 hour in 37°C and 5% CO_2_. The inoculant was removed and replaced with overlay medium containing 1% Aquacide II (Sigma-Aldrich) supplemented with 2% FBS, 1% antibiotic/antimycotic, and 2 mM of l-glutamine (Gibco-Thermo Fisher Scientific) and incubated at 37°C under 5% CO_2_ for three days. The cells were fixed with 3.7% formaldehyde (Sigma-Aldrich) and stained with 2% crystal violet (Sigma-Aldrich).

### 2.2. Active Compounds

The [6]-gingerol ((*S*)-5-hydroxy-1-(4-hydroxy-3-methoxyphenyl)-3-decanone) (Sigma-Aldrich, GI046) was dissolved in 100% dimethyl sulfoxide (DMSO) (Applichem CAS67-68-5) to a final concentration of 20 mM and stored in -20°C according to manufacturer's instruction. Ribavirin (Sigma-Aldrich, R9644) was used as a positive control at 2.6 *μ*g/ml concentration, as demonstrated by Franco et al. [25]. The compound was dissolved in 100% DMSO (Applichem CAS67-68-5), resulting in a stock concentration of 10 mg/ml, and stored at -20°C according to manufacturer's instruction. Both compounds were diluted to working concentration with complete RPMI medium. The highest final concentration of 0.75% DMSO in the working concentration (used in 0.15 mM [6]-gingerol dilution) was included as a vehicle control.

### 2.3. Cell Cytotoxicity Assay

Cytotoxicity of [6]-gingerol to HepG2 was measured by a cell viability assay performed using the classical 3-(4,5-dimethyl-thiazol-2-yl)-2,5-diphenyltetrazolium bromide (MTT) (Vybrant-Thermo Fisher Scientific) assay. HepG2 were seeded 1 × 10^5^ cells/well in 96-well plates and incubated overnight. The cells were challenged with medium, vehicle, or various concentrations of [6]-gingerol at 37°C and 5% CO_2_. After 48 hours incubating, the medium was removed and replenished with 100 *μ*l fresh medium. The cell viability assay was then performed according to manufacturer's instruction. Briefly, 10 *μ*l of 12 mM MTT stock was added to wells containing cells and then incubated at 37°C for 2 hours. After incubation, 100 *μ*l of the 10% SDS in 0.01 M HCl solution was added, followed by overnight incubation at 37°C. Absorbance from each well was measured at 570 nm using a microplate reader.

The article "[6]-Gingerol Inhibits Chikungunya Virus Infection by Suppressing Viral Replication" was published in 2021. Journal: Biomed Res Int.

### 2.4. Virucidal Assay

We performed a virucidal assay to examine direct virucidal activity of [6]-gingerol against CHIKV, modified from Ahmad et al. [26]. Approximately 2 × 10^5^ PFU of CHIKV-JMB-192 was incubated directly with medium, vehicle, ribavirin, or various concentrations of [6]-gingerol (0.05 mM, 0.1 mM, and 0.15 mM) at 37°C for 1 hour, after which infectious virus titer was determined by standard plaque assay. This was done in triplicate.

### 2.5. Antiviral Activity of [6]-Gingerol

Four different treatments were assayed to examine the indirect antiviral activity of [6]-gingerol: pre-, post-, full-, and prevention assay. Treatment was applied to 2 × 10^5^ HepG2 cells/well seeded in 24-well plates, which had been incubated at 37°C and 5% CO_2_ overnight. CHIKV-JMB-192 strain was used for infection with multiplicity of infection/MOI = 1.0.

In pretreatment assay, CHIKV was pretreated with medium, vehicle, ribavirin, or various concentrations of [6]-gingerol at 37°C for 1-hour preceding addition to HepG2 at 37°C and 5% CO_2_ for 1 hour. The cells were washed and replenished with medium only following 48 hours of incubation at 37°C and 5% CO_2_. In posttreatment, CHIKV was added to HepG2 cells for 1 hour at 37°C and 5% CO_2_. After washing, the cells were treated with medium, vehicle, ribavirin, or various concentrations of [6]-gingerol and incubated at 37°C and 5% CO_2_ for 48 hours. Full treatment was a combination of pre- and posttreatments. In the prevention assay, HepG2 cells were treated with medium, vehicle, ribavirin, or various concentrations of [6]-gingerol at 37°C and 5% CO_2_ for 1 hour before being infected with CHIKV at 37°C and 5% CO_2_ for 1 hour. After washing, the cells were supplemented with fresh medium and incubated at 37°C and 5% CO_2_ for 48 hours. In all treatments, the supernatant was collected after 48 hours of incubation, as shown in Turnip et al. [27], and measured for viral titers by standard plaque assay.

The article "[6]-Gingerol Inhibits Chikungunya Virus Infection by Suppressing Viral Replication" was published in 2021. Journal: Biomed Res Int.

### 2.6. Statistical Analysis

All statistical analysis was done using the SPSS Statistics program (Ver. 24), and the two-tailed *t*-test for independent samples was used. A *p* value of less than 0.05 was considered as statistically significant. The 50% cytotoxic concentration (CC_50_) and 50% inhibitory concentration (IC_50_) values were determined with AAT Bioquest QuestGraph™ IC_50_ calculator (https://www.aatbio.com/tools/ic50-calculator). The selectivity index was calculated by dividing CC_50_ by IC_50_.

## 3. Results

### 3.1. Cytotoxicity of [6]-Gingerol

The MTT assay was used to determine the cytotoxicity of [6]-gingerol in HepG2 cells. The 50% cytotoxic concentration (CC_50_) of [6]-gingerol was measured at 0.21 mM. No significant cytotoxicity was observed for cells treated with vehicle control (0.75% DMSO) (Figure 2(a)), which was the highest final concentration of the solvent used to dissolve [6]-gingerol in cell culture media. Morphologic observation also showed that HepG2 cells treated with ≤0.2 mM [6]-gingerol were healthy with minimal cell death. However, the cells treated with >0.2 mM [6]-gingerol (0.4 mM, 0.5 mM, and 1.0 mM) gradually suffered cell death as the concentration increased (Figure 2(b)). The cell death was particularly significant at 1.0 mM [6]-gingerol as almost all the cells were dead.

### 3.2. Evaluation of Virucidal Activity of [6]-Gingerol

To examine virucidal activity of [6]-gingerol, CHIKV was incubated at 37°C with medium only, vehicle, ribavirin, or various concentrations of [6]-gingerol for 1 hour. Upon incubation, virus viability and titer were determined by plaque assay. As presented in Figure 3, [6]-gingerol showed limited virucidal activity in a dose-dependent manner. At a low concentration (0.05 mM), almost no virucidal activity of [6]-gingerol was observed. A reduction of viral titer was only observed at higher concentrations (0.1 mM and 0.15 mM) with less than 1 log_10_ (or around 30%) viral reduction at the highest concentration tested. The measured IC_50_ was 0.24 mM for virucidal activity in comparison to untreated medium control. Ribavirin also showed relatively weak virucidal activity with approximately 20% reduction of viral titer.

### 3.3. [6]-Gingerol Inhibits CHIKV Replication in Post- and Full-Treatment Assays

To identify the indirect antiviral activity of [6]-gingerol and its mechanism, we employed four different assays: pre-, post-, full-, and prevention assays. Antiviral activity was observed in post- and full-treatment assay, even at the lowest concentration tested (Figure 4). At 0.05 mM, [6]-gingerol significantly reduced approximately 75% of viral titer. At higher concentrations (0.1 mM and 0.15 mM), more than 95% viral reduction was achieved. The findings indicate that [6]-gingerol effectively inhibits CHIKV infection by suppressing viral replication. The measured IC_50_ for both assays were 0.038 mM and 0.031 mM for post- and full-treatment assay, respectively, which were much lower than the observed CC_50_. The selectivity index indicates a value around 5 and 8 for the post- and full treatment, respectively.

The article "[6]-Gingerol Inhibits Chikungunya Virus Infection by Suppressing Viral Replication" was published in 2021. Journal: Biomed Res Int.

## 4. Discussion

Although CHIK has a lower fatality rate compared to similar arboviral disease such as dengue, the daily life of an infected person is greatly affected as the joint pain remains for quite a long period. Therefore, the development of CHIKV antiviral agents needs to target a significant reduction of viral load in order to prevent the debilitating effects caused by the immune response. Secondary metabolites may serve as prospective antiviral agents since many of them have been proven to effectively treat the disease with additional benefits. Ginger has been used as a herbal remedy for generations, especially in Asian countries. Due to its widely known various health benefits, we examined the antiviral activity of [6]-gingerol, one of the main bioactive compounds of ginger against CHIKV. We used the wild-type CHIKV circulating in Indonesia as challenge virus which has been characterized as Asian genotype [6]. Currently, this genotype is the predominant CHIKV genotype in Indonesia, making up more than ninety percent of cases [4].

In this study, we used the HepG2 cell line for cytotoxicity, virucidal, and antiviral assays. For *in vitro* study, HepG2 has been proven to have a high susceptibility to CHIKV infection [28]. Therefore, this cell line has been used in CHIKV antiviral studies [29, 30]. With regard to CHIK pathogenesis in humans, CHIKV was also reported to disseminate to the liver after replication in the skin [7]. Hence, using the HepG2 cell line may help mimic the CHIKV pathogenesis in humans.

We examined the cytotoxicity of [6]-gingerol in the HepG2 cell line. The CC_50_ of [6]-gingerol in HepG2 after a 48 hr incubation was 0.21 mM. Morphologically, the cells challenged with [6]-gingerol at concentrations less than the CC_50_ were healthy with minimal cell death, confirming the CC_50_ concentration. The same cytotoxicity study using different cell lines showed half of our CC_50_ value (0.1 mM, 0.102 mM, and 0.102 mM for HCT15, L929, and RAW264.7, respectively) when treated for 24 hours [31]. This might be caused by the shorter incubation period and the different cell lines used. In our study, we treated the cells for 48 hours since the CHIKV infection in HepG2 cells was maximized after 48 hours of incubation, as shown in our previous study [27].

The article "[6]-Gingerol Inhibits Chikungunya Virus Infection by Suppressing Viral Replication" was published in 2021. Journal: Biomed Res Int.

We examined the direct virucidal activity of [6]-gingerol against CHIKV. As presented in Figure 3, [6]-gingerol showed limited virucidal activity. Inhibition of viral activity was only observed at higher concentrations (0.1 mM and 0.15 mM) with less than 1 log_10_ PFU/mL viral reduction. Virucidal compounds inhibit viral activity by inactivating extracellular viral particles or by penetrating virions and destroying the viral genome [26]. As a control, ribavirin showed virucidal activity, although relatively little, which was also observed elsewhere [32, 33].

As [6]-gingerol only showed relatively limited direct virucidal activity against CHIKV, we examined the indirect antiviral activity of the compound in HepG2 cells. We employed four indirect antiviral assays. The pretreatment assay was designed to identify the ability of [6]-gingerol to block virus entry to host cells during infection while the posttreatment assay examined the ability of [6]-gingerol to inhibit viral replication within CHIKV-infected cells. The full-treatment assay, a combination of pre- and posttreatment assays, examined the full antiviral capacity of [6]-gingerol against CHIKV. The prevention assay monitored protective effect of [6]-gingerol treatment to the host cells preceded CHIKV infection.

From the four assays employed, antiviral activity was observed in the post- and full-treatment assays, indicating that [6]-gingerol effectively inhibits viral replication after CHIKV infects the cells. The IC_50_ were 0.038 mM and 0.031 mM for post- and full-treatment assays, respectively, which were much lower than the CC_50_. The selectivity index (SI) is an important indicator to identify the promising antiviral activity of a compound with negligible toxicity. Theoretically, a higher SI indicates the effectiveness and safety of the compound. Here, we found the selectivity index of [6]-gingerol was 5 and 8 for the post- and full treatments, respectively. Although these SIs were not very high, they indicate that [6]-gingerol has the potential to treat CHIKV infection. For comparison, the reduction of viral load by [6]-gingerol was significantly higher than ribavirin.

Several studies have reported on the antiviral activity of fresh ginger, ginger extract, or other processed forms of ginger through various modes of action. Ginger essential oil was reported to have direct antiviral activity against herpes simplex virus type 2 [34]. Influenza virus H9N2 replication was inhibited by aqueous extract of ginger *in vitro* [35]. Fresh ginger was reported to inhibit human respiratory syncytial virus activity by blocking viral attachment and internalization [36]. Together, these findings indicate that the compound behaves differently depending on the pathogen.

The article "[6]-Gingerol Inhibits Chikungunya Virus Infection by Suppressing Viral Replication" was published in 2021. Journal: Biomed Res Int.

Understanding the mechanism of action of antiviral compounds is an important step in drug development which helps their evaluation and application in disease treatment. In this study, we observed that the antiviral mechanism of [6]-gingerol was the inhibitory effect on CHIKV replication after the virus infects host cells. Similar antiviral mechanisms have been reported. Harringtonine, a cephalotaxine alkaloid, inhibited CHIKV replication in the early stages which occurred after viral entry into cells [37]. Several flavonoids were also reported to inhibit CHIKV replication at postentry stage, including silymarin, hesperitin, and naringenin [38, 39]. However, different antiviral mechanisms were also observed with different compounds. For example, curcumin inhibited binding of viruses to the cells during CHIKV infection [40]. Therefore, the antiviral mechanism seems to be very specific for each compound. Regarding its weak virucidal activity, inhibition of CHIKV replication at posttreatment by [6]-gingerol indicates an important role in host defensive mechanisms. Practically, inhibition of viral replication is more applicable for CHIK treatment since it allows the antiviral drug to be administered after someone is infected with CHIKV rather than as a supplement that is consumed before infection occurs.

## 5. Conclusion

This study was the first to report the antiviral activity of [6]-gingerol against CHIKV and its possible mechanism of action. Considering the substantial public and economic impact of CHIKV infection due to the prolonged persisting arthralgia, this study provides insight into the potential use of [6]-gingerol as an antiviral agent for CHIKV infection. Further studies are encouraged to establish effective strategies to utilize [6]-gingerol for CHIK treatment.

## Figures and Tables

**Figure 1:** The chemical structure of 6-gingerol (source: http://chemspider.com/Chemical-Structure.391126.html).

**Figure 2:** Determination of [6]-gingerol cytotoxicity in HepG2 cells by MTT assay. (a) HepG2 cells were incubated with medium, vehicle, or [6]-gingerol (0.1 mM, 0.2 mM, 0.4 mM, 0.5 mM, and 1.0 mM) for 48 hours followed by MTT cell viability assay. Data derived from triplicates. (b) Morphology of HepG2 cells after 48 hours of incubation with medium or [6]-gingerol.

**Figure 3:** Evaluation of virucidal activity of [6]-gingerol against CHIKV. CHIKV-JMB-192 was incubated directly with medium, vehicle, ribavirin, or [6]-gingerol (0.05 mM, 0.1 mM, and 0.15 mM) at 37°C and 5% CO_2_ for 1 hour. Virus titer was determined by standard plaque assay. Data derived from triplicates.

The article "[6]-Gingerol Inhibits Chikungunya Virus Infection by Suppressing Viral Replication" was published in 2021. Journal: Biomed Res Int.

**Figure 4:** Evaluation of antiviral activity of [6]-gingerol upon CHIKV infection in HepG2 cells. Antiviral activity of [6]-gingerol was evaluated in pre-, post-, full-, and prevention treatment cell modes. Viral titer was measured by standard plaque assay. Statistical significance was determined using two-tailed *t*-test for independent samples (^∗^*p* < 0.01 and ^∗∗^*p* < 0.001).

## Data Availability

The antiviral data used to support the findings of this study are included within the article.
